# Oxidative Stress and Mitochondrial Functions in the Intestinal Caco-2/15 Cell Line

**DOI:** 10.1371/journal.pone.0011817

**Published:** 2010-07-27

**Authors:** Rame Taha, Ernest Seidman, Genevieve Mailhot, François Boudreau, Fernand-Pierre Gendron, Jean-François Beaulieu, Daniel Ménard, Edgard Delvin, Devendra Amre, Emile Levy

**Affiliations:** 1 Department of Nutrition, Research Center, CHU-Sainte-Justine, Université de Montréal, Montreal, Canada; 2 Research Institute, McGill University, Montreal, Canada; 3 Canadian Institutes for Health Research Team on the Digestive Epithelium, Department of Anatomy and Cellular Biology, Faculty of Medicine and Health Sciences, Université de Sherbrooke, Sherbrooke, Canada; 4 Department of Biochemistry, Research Center, CHU-Sainte-Justine, Université de Montréal, Montreal, Canada; 5 Department of Pediatrics, Research Center, CHU-Sainte-Justine, Université de Montréal, Montreal, Canada; New Mexico State University, United States of America

## Abstract

**Background:**

Although mitochondrial dysfunction and oxidative stress are central mechanisms in various pathological conditions, they have not been extensively studied in the gastrointestinal tract, which is known to be constantly exposed to luminal oxidants from ingested foods. Key among these is the simultaneous consumption of iron salts and ascorbic acid, which can cause oxidative damage to biomolecules.

**Methodology/Principal Findings:**

The objective of the present work was to evaluate how iron-ascorbate (FE/ASC)-mediated lipid peroxidation affects mitochondrion functioning in Caco-2/15 cells. Our results show that treatment of Caco-2/15 cells with FE/ASC (0.2 mM/2 mM) **(1)** increased malondialdehyde levels assessed by HPLC; **(2)** reduced ATP production noted by luminescence assay; **(3)** provoked dysregulation of mitochondrial calcium homeostasis as evidenced by confocal fluorescence microscopy; **(4)** upregulated the protein expression of cytochrome C and apoptotic inducing factor, indicating exaggerated apoptosis; (5) affected mitochondrial respiratory chain complexes I, II, III and IV; (6) elicited mtDNA lesions as illustrated by the raised levels of 8-OHdG; (**7**) lowered DNA glycosylase, one of the first lines of defense against 8-OHdG mutagenicity; and (8) altered the gene expression and protein mass of mitochondrial transcription factors (mtTFA, mtTFB1, mtTFB2) without any effects on RNA Polymerase. The presence of the powerful antioxidant BHT (50 µM) prevented the occurrence of oxidative stress and most of the mitochondrial abnormalities.

**Conclusions/Significance:**

Collectively, our findings indicate that acute exposure of Caco-2/15 cells to FE/ASC-catalyzed peroxidation produces harmful effects on mitochondrial functions and DNA integrity, which are abrogated by the powerful exogenous BHT antioxidant. Functional derangements of mitochondria may have implications in oxidative stress-related disorders such as inflammatory bowel diseases.

## Introduction

Reactive Oxygen Species (ROS) are by-products of normal aerobic metabolism and are now considered to be important signaling molecules that play a role in gene expression, cell growth and survival as well as oxygen sensing in various cell types [1], [2]. The generation of ROS by a cascade of reactions is efficiently blocked by various endogenous antioxidants to overcome their potentially injurious actions [2], [3]. However, excessive formation of ROS leads to lasting oxidative stress, characterized by an imbalance between oxidant-producing systems and antioxidant defense mechanisms, which can trigger cell damage by oxidizing macromolecular structures (lipids, proteins and DNA) and modifying their biological functions that ultimately causes cell death [4]. Thus, depending on their cell concentrations, ROS can act as either beneficial or harmful biological agents.

The gastrointestinal tract is frequently exposed to noxious stimuli that may cause oxidative stress and injury. In fact, oxygen free radicals are generated both in the lumen and in the intestinal mucosa. Intraluminal pro-oxidants from ingested nutrients, such as alcohol, cholesterol oxides or iron salts and ascorbic acid, frequently consumed together in multiple-vitamin preparations or ingested foods, can build a pro-oxidant milieu [5]–[7]. Moreover, local microbes or infections, ischemia/reperfusion, gastric acid production and non-steroidal anti-inflammatory drugs may promote the formation of reactive radicals [8]–[10]. In addition, the influx of leukocytes, neutrophils and monocytes (associated with inflammation) can produce further ROS via respiratory burst enzymes as well as those involved in prostaglandin and leukotriene metabolism [11]. Clearly, significant oxidative stress has been said to be always associated with mucosal erosions and a causative role in a variety of gastrointestinal diseases such as Crohn's disease and ulcerative colitis [12]–[14].

Despite the frequent occurrence of oxidative stress in the gastrointestinal tract and its involvement in the initiation and propagation of the chronic inflammatory response in chronic bowel diseases [15], little is known about mitochondrion response even though this special organelle is both a major source of oxidants and a target for their damaging effects [16]. We have hypothesized that oxidative stress may affect various mitochondrial functions, including ATP production, calcium (Ca^2+^) homeostasis, cellular redox state regulation, apoptosis, as well as mtDNA integrity [17], [18]. Therefore, the specific aim of the present study was to characterize the interplay between oxidative stress and mitochondrial dysfunction in the Caco-2/15 cell line using the iron-ascorbate (FE/ASC) oxygen radical-generating system, which participates in lipid peroxidation in inflammatory bowel diseases (IBD) and represents a powerful tool in our hands for the initiation of highly reactive hydroxyl radicals and for the down-regulation of endogenous antioxidants [19]–[26].

## Materials and Methods

### Caco-2/15 Cell Cultures

The colon carcinoma cell line, Caco-2/15 (ATCC, Rockville, MD), was cultured at subconfluent stages in MEM (GIBCO-BRL, Grand Island, NY) containing 1% penicillin-streptomycin and 1% MEM non-essential amino acids (GIBCO-BRL) and supplemented with 10% decomplemented fetal bovine serum (FBS) (Flow, McLean, VA) as described previously [27]. Briefly, Caco-2/15 cells (passage 20-30) were maintained in T-75-cm^2^ flasks (Corning Glass Works, Corning, NY). Cultures cells were split (1∶6) when they reached 90% confluence by use of 0.05% trypsin-0.5 mM EDTA (GIBCO-BRL). For individual experiments, cells were plated at a density of 1×10^6^ cells/well on 24.5 mm polyester Transwell filter inserts with 0.4-µm pores (Coster, Cambridge, MA) in MEM supplemented with 5% FBS. Cells were cultured for 21 days post confluence, at which the Caco-2/15 cells are highly differentiated and appropriate for lipid synthesis and metabolism. The medium was refreshed every second day. To determine the implication of oxidative stress *per se* in alterations in mitochondrial functions, Caco-2/15 cells were incubated with FE/ASC (0.2 mM/2 mM) for 6 h alone and/or with the antioxidant butylated hydoxytoluene (BHT) (2,6-di-*t*-butyl-*p*-cresol, Sigma, St-Louis, MA) (50 µM). Caco-2/15 cells were divided into four groups: control (without any addition), oxidative (FE/ASC), antioxidant (BHT), oxidative and antioxidant (FE/ASC + BHT).

### Lipid Peroxidation

Caco-2/15 cells were cultured in the presence or absence of (0.2 mM/2 mM) FE/ASC added to the medium. Incubation periods were terminated with 50 µM BHT to measure malondialdehyde (MDA). The level of MDA formed during the oxidative reaction was determined by HPLC, as previously described [19]. Briefly, proteins were first precipitated with a 10% sodium tungstate (Na_2_WO_4_) (Aldrich, Milwaukee, WI) solution. The protein-free supernatants were then reacted with an equivalent volume of 0.5% (wt/vol) thiobarbituric acid solution (TBA; Sigma) at 90°C for 60 min. After cooling to room temperature, the pink chromogene [(TBA) 2-MDA] was extracted with 1-butanol and dried over a stream of nitrogen at 37°C. The dry extract was then resuspended in a potassium dehydrogen phosphate (KH_2_PO_4_)/methanol mobile phase (70; 30, pH 7.0) before MDA determination by HPLC with fluorescence detection.

### Assessment of Intracellular ATP

Intracellular ATP was measured by luciferase driven bioluminescence using ATP Bioluminescence Assay Kit from (Calbiochem, EMD Chemicals, Inc. Gibbstown, NJ) as reported previously [28]. Values were then normalized further with regard to the protein content of the respective sample. All Caco-2/15 culture cells were performed in duplicate.

### Calcium Measurements by Confocal

For mitochondrial Ca^2+^ monitoring, Caco-2/15 cells were trypsinized, transferred from cell culture flasks to 8-well chamber slides (Lab-Tek™ Nunc, Rochester, NY) at a density of 2,5×10^4^ cells in 500 µl of cell culture medium. After a period of three days, cells were serum-starved and incubated with FE/ASC and/or BHT as described above. Cells were rinsed twice in serum-free culture medium and loaded with a mixture of 5 µM Rhod-2/AM (Molecular Probes, Eugene, OR), a fluorescent probe specific for mitochondrial Ca^2+^, with 0,01% pluronic acid for 30 min at 37°C as described previously [29]–[31]. Medium was removed, replaced with dye-free culture medium and incubated for an additional 60 minutes at 37°C. Thereafter, 1 µl of the fluorescent mitochondria-specific dye MitoTracker™ (green fluorescence, Molecular Probes) was added to each well at the last 30 min of incubation. Cells were visualized using an inverted laser-scanning confocal microscope equipped with a 40× objective (LSM 510, Zeiss). Excitation wavelength was 488 nm and fluorescence emission was recorded at 543 nm (for Rhod-2) and 516 nm (for MitoTracker™). Six to eight fluorescence images were randomly chosen in selected microscopic fields. Fluorescence intensity was quantified using the Image J software (http://rsb.info.nih.gov/ij).

### Mitochondrial Preparations

Mitochondria were isolated using standard differential centrifugation techniques [32]. Briefly, Caco-2/15 cells were treated with (0.2 mM/2 mM) FE/ASC and/or (50 µM) BHT for 6 h at 37°C. Cells were homogenized with a glass pestle Dounce homogenizer in a buffer containing 210 mM mannitol, 70 mM sucrose, 1 mM EGTA, 0.5% fatty acid-free bovine serum albumin, and 5 mM HEPES, pH 7.2. The homogenate was centrifuged at 1000 x *g* for 10 min at 4°C. The supernatant was then collected and centrifuged at 10000 x g for 10 min to obtain the pellets containing mitochondria. The pellets were used immediately or stored at −80°C. The protein contents of mitochondrial suspension were determined by the Bradford assay (BioRad, Mississauga, ON) with BSA as a standard.

### Evaluation of 8-hydroxy -2-deoxyguanosine

Oxidative DNA damage in whole Caco-2/15 cells, nuclei and mitochondria was evaluated by assessing 8-hydroxy -2-deoxyguanosine (8-OHdG) with high-sensitivity competitive ELISA assays performed with a commercial kit from Genox Corporation (Baltimore, USA). Briefly, 8-OHdG antibody plus sample DNA were added to a 96-well plate percolated with 8-OHdG and incubated overnight at 4°C. After the plate was washed, horseradish peroxidase–conjugated secondary antibody was added for 1 h at room temperature. After washing, 3,3′,5,5′-tetramethylbenzidine was added and incubated for 15 min at room temperature in the dark. The reaction was terminated by the addition of phosphoric acid, and absorbance was measured at 450 nm. All assays were performed in duplicate. Negative controls and 8-OHdG standards (0.125–10 ng/mL) were included in the assay. The average concentration of 8-OHdG was calculated for each sample based on the standard curve.

### Mitochondrial Enzyme Assays

The activities of respiratory chain complexes were assayed as previously described in detail [32]–[34]. Briefly, 20–30 µg of mitochondrial protein were used for each complex every 30 sec for 5 min. The activity of complex I (NADH: ubiquinone oxidoreductase) was measured by monitoring the reduction of decylubiquinone. Complex II (succinate:ubiquinone oxidoreductase) activity was examined by monitoring the reduction of dichloroindophenol when coupled to complex II-catalyzed reduction of decylubiquinone. Complex III (ubiquinol:ferricytochrome C oxidoreductase) activity was assayed using oxidized cytochrome C. The activity of complex IV (cytochrome C oxidase) was determined by oxidation of reduced cytochrome C. Enzyme activities were expressed in nanomoles of substrate used per minute per milligram of protein. Enzyme assays for all complexes were performed in duplicate in mitochondrial fraction of Caco-2/15 cell line. Complex I, II, III, IV chemicals were purchased from Sigma Chemical, St Louis, MO.

### Western Blots

To assess the protein mass of mitochondrial transcription factors (mt TF): mtTFA, mtTFB1, mtTFB2 and POLRMT, as well as 8-oxoG-DNA glycosylase (OGG1), apoptosis-inducing factor (AIF) and cytochrome C, Caco-2/15 cells were homogenized and adequately prepared for Western blotting as described previously [22], [23], [27], [35]–[39]. The Bradford assay (Bio-Rad) was used to estimate protein concentration. Proteins were denatured in sample buffer containing SDS and β-mercaptoethanol, separated on a 4–20% gradient SDS-PAGE and electroblotted onto nitrocellulose membranes. Nonspecific binding sites of the membranes were blocked with defatted milk proteins followed by the addition of primary antibodies directed against the different proteins. The relative amount of primary antibody was detected with species-specific horseradish peroxidase-conjugated secondary antibody. Even though identical protein amounts of tissue homogenates were applied, the β-actin protein was used to confirm equal loading on SDS-PAGE (results not shown). Blots were developed and the mass of proteins was quantitated using an HP Scanjet scanner equipped with a transparency adapter and software. Rabbit polyclonal mtTFA Ab was obtained from Santa Cruz Biotechnology Santa Cruz, CA; rabbit polyclonal POLRMT from Abcam, Cambridge, MA; and mouse polyclonal mtTFB1 and mtTFB2 Ab, rabbit polyclonal OGG1 Ab, rabbit polyclonal AIF Ab, and mouse monoclonal cytochrome C Ab from Novus Biologicals, Inc.

### RT-PCR

Experiments for mRNA quantification as well as for GAPDH (as a housekeeping gene) were performed in Caco2/15 cells using the UNO II thermocycler (Biometra) as reported previously [35], [40]. Approximately 30–40 cycles of amplification were used at 95°C for 30 s, 58°C for 30 s, and 72°C for 30 s. Amplicons were visualized on standard ethidium bromide-stained agarose gels. Under these experimental conditions related to RT-PCR, the cycles for mtTFA, mtTFB1, mtTFB2, POLRMT, OGG1 and GAPDH were 31, 31,35,31,31, and 30, respectively corresponding to the linear portion of the exponential phase. Fold induction and quantification were determined with the software UN-SCAN-IT gel 6.1.

### Primers Used

**GAPDH** ( **F-** AGAAGGCTGGGGCTCATT/**R**-GGGCCATCCACAGTCTTCT)

**H-OGG1 (** **F**-GGGGATTCACAAGGTGAAGA/**R**-GTAAGCTGGCTTGCATCACA)

**POLRMT (** **F**-CATCACCTACACCCACAACG/**R**-GTGCACAGAGACGAAGGTCA)

**H-mtTFB2 (** **F**-GTCGCTTTTGCATTTTAGGG/**R**-GCTGTCCAAGGAACTGCTTC)

**h-mtTFB1** ( **F**-CTCCTGGACTTGAGGCTGAC/**R**-TTCTCAGTTTCCCAGGTGCT)

**h-mtTFA (** **F**-GGGTTCCAGTTGTGATTGCT/R-TGGACAACTTGCCAAGACAG)

### Statistical Analyses

Statistical analyses of data were performed with Prism 4.03 software (GraphPad Software). All values were expressed as the mean ± SEM. The data were evaluated by ANOVA, where appropriate, and the differences between the means were assessed using the Bonferroni's multiple comparison test. A *p*-value of less than 0.05 was considered to be significant.

## Results

### MDA Generation after Iron-Ascorbate Exposure

Before evaluating the role of oxidative stress on mitochondrial function, we evaluated the effectiveness of FE/ASC in initiating lipid peroxidation after incubation with Caco-2/15 cells. At the end of a 6-h culture period, the degree of lipid peroxidation was determined by measuring MDA in cells. As illustrated in Figure 1, FE/ASC induced a significant increase in MDA levels above baseline values compared with control cells. The concentration of MDA was 4-fold higher in cells supplemented with FE/ASC compared with untreated cells. Pre-incubation with the strong antioxidant BHT markedly suppressed the production of MDA, providing direct evidence for the ability of the FE/ASC system to provoke profound lipid peroxidation.

**Figure 1:** Malondialdehyde (MDA) concentrations in Caco-2/15 cells challenged with iron/ascorbate and/or BHT. At 21 days of differentiation, cells were exposed to (0.2 mM/2 mM) FE/ASC, (50 µM) BHT or both for 6 h at 37°C. Oxidative stress was assessed by measuring MDA as an index of lipid peroxidation. Values are means ± SEM for three independent experiments. ^*^P<0.05.

### Effect of FE/ASC on Cellular ATP Content

The main function of the mitochondrion is the production of energy in the form of ATP via oxidative phosphorylation and oxygen consumption. We therefore assessed the amount of ATP levels in Caco-2/15 cells exposed to the FE/ASC oxygen radical-generating system. As noted in Figure 2, the administration of FE/ASC led to a four-fold reduction compared with untreated cells. Moreover, pre-incubation with BHT at a concentration of 0.5 mM resulted in a trend of ATP normalization.

**Figure 2:** ATP Levels in Caco-2/15 cells exposed to iron/ascorbate in the presence or absence of BHT. Caco-2/15 cells were grown on 96-well plates and, after 21 days post confluence, they were treated with (0.2 mM/2 mM) FE/ASC and/or (50 µM) BHT for 6 h at 37°C. ATP levels were measured with a bioluminescence assay and corrected for intracellular protein concentrations. Values are expressed as ng of ATP per µg of cellular protein and represent the means ± SEM for three independent experiments. ^*^P<0.001.

### Oxidative Phosphorylation Activity

Since mitochondrial oxidative phosphorylation (OXPHOS) is fundamental to all aspects of cell life under aerobic conditions, we evaluated its activity during oxidative stress. The enzymatic activity related to complexes I, II, III, and IV was performed on mitochondrial fraction prepared from Caco-2/15 cells. Our findings documented a significant decrease in the specific activities of complex I, II, III and IV following FE/ASC treatment (Figure 3). Pre-incubation with BHT abrogated the decline in the OXPHOS enzymatic activities.

**Figure 3:** Effect of iron/ascorbate and/or BHT treatment on enzymatic activities of mitochondrial respiratory chain complexes in Caco-2/15 cells. Enzyme activities of mitochondrial respiratory chain complexes I, II, III, IV were measured by spectrophotometric assays in mitochondrial samples in Caco-2/15 cells treated with (0.2 mM/2 mM) FE/ASC and/or (50 µM) BHT for 6 h at 37°C. Enzyme activities are expressed as nmol/min/mg protein. Each value represents the mean ± SEM for 3 separate experiments performed in duplicate. *P<0.05 vs. controls.

### Changes in Mitochondrial Calcium Induced by Iron-Ascorbate in Caco-2/15 Cells

We next tested whether FE/ASC caused a change in mitochondrial Ca^2+^ in Caco-2/15 cells using the positively charged and cell permeant Ca^2+^ indicator, Rhod-2/AM, which accumulates predominantly in the negatively charged matrix of the mitochondria. The dye Mitotracker™ was used to confirm the mitochondrial localization of Rhod-2. As presented in Figure 4D, FE/ASC treatment of Caco-2/15 cells induced an increase in Rhod-2 fluorescence that appears predominantly located in the mitochondria as demonstrated by the yellow spots of strong intensity found in the merged image (Figure 4F). In contrast, the distribution pattern of colocalized Rhod-2 and Mitotracker™ observed in control cells revealed spots of less intensity characterized by a more diffuse distribution (Figure 4E). Quantification of Rhod-2 fluorescence intensity is shown in Figure 5. Cells exhibited an increase in Rhod-2 fluorescence after FE/ASC treatment whereas pre-incubation with BHT restored fluorescence intensity to control level.

**Figure 4:** Influence of oxidative stress on mitochondrial calcium homeostasis in Caco-2/15 cells. Representative fluorescence images of control and FE/ASC-treated Caco-2/15 cells loaded with the mitochondrial dye MitoTracker™ (**A, B**) and the mitochondrial Ca^2+^ indicator Rhod-2 (**C, D**). Merged images (**E, F**) indicate colocalization of the two dyes in the mitochondria. Mitochondrial Ca^2+^ accumulation is visible upon oxidative stress (**arrow**). Scale bar-10 µm.

**Figure 5:** Quantification of Rhod-2 fluorescence intensity in Caco-2/15 Cells subjected to iron/ascorbate and/or BHT treatment. Caco-2/15 cells pretreated for 6 h with (0.2 mM/2 mM) Fe/ASC and/or (50 µM) BHT were loaded with 5 µM of Rhod-2 AM for 30 minutes at 37°C. Fluorescence intensity was quantified by image analysis as described in Material and Methods. Six to eight fluorescence images from three independent experiments were randomly chosen. Results were calculated by dividing the pixel intensity by the area of the spot (µm^2^). Data illustrated represent the means ± SEM. ^*^P<0.001.

### AIF and Cytochrome C Protein Expression

AIF is normally located in the inter-membrane space of mitochondria and is involved in initiating a caspase-independent pathway of apoptosis by causing DNA fragmentation and chromatin condensation. Furthermore, when cell death is triggered by an apoptotic stimulus, cytochrome C is released into the cytosol, and contributes to the caspase-dependent pathway of apoptosis. Western blot analysis revealed a marked (P<0.001) increase in the level of AIF and cytochrome C protein mass in Caco-2/15 cells following FE/ASC compared with controls (Figures 6). Pre-incubation with BHT before the addition of FE/ASC prevented the rise in AIF and cytochrome C protein mass.

**Figure 6:** Cytochrome C and AIF expression levels in Caco-2/15 Cells treated with iron/ascorbate and/or BHT. Caco-2/15 cells were incubated with (0.2 mM/2 mM) FE/ASC and/or (50 µM) BHT for 6 h at 37°C. Gene and protein expression were determined by RT-PCR and Western blotting, respectively. Values are expressed as means ± SEM for three independent experiments. ^*^P<0.001.

### Quantification of Oxidative DNA Damage in Caco-2/15

ELISA for 8-OHdG, a recognized marker of oxidative DNA damage, was used to quantify oxidative DNA damage in Caco-2/15 cells. Figure 7 shows the average concentration of 8-OHdG detected in the control and experimental groups. Results clearly indicate that the level of oxidative DNA damage in mitochondria was significantly (P<0.001) higher in Caco-2/15 exposed to FE/ASC-mediated lipid peroxidation (Figure 7A). The oxidative DNA damage was attenuated after pre-incubation with BHT. On the other hand, no significant changes were noted in the homogenate or nucleus (Figure 7B and 7C).

**Figure 7:** Influence of iron/ascorbate treatment in the presence of absence of BHT on 8-hydroxy -2-deoxyguanosine level in Caco-2/15 cells. The levels of 8-hydroxy -2-deoxyguanosine (8-OHdG) were measured by ELISA kit assay in (A) mitochondrial, (B) homogenate and (C) nucleus samples in Caco-2/15 cells treated with (0.2 mM/2 mM) FE/ASC and/or (50 µM) BHT for 6 h at 37°C. Values are means ± SEM for three independent experiments. ^*^P<0.001.

### OGG1 Repair Enzyme Level

In mitochondria, the base excision repair pathway is primarily responsible for removing 8-OHdG from DNA [41]. In humans, 8-oxodG is repaired by 8-oxoguanine DNA glycosylase (OGG1), an enzyme that recognizes and hydrolyzes the aberrant base from the DNA backbone. We, therefore, examined its gene expression and protein mass in Caco-2/15 cells. As well illustrated in Figure 8, treatment with FE/ASC resulted in a significant (P<0.001) reduction of OGG1 mRNA and protein mass compared with controls. However, pre-incubation of Caco-2/15 cells with BHT prevented the decline in OGG1 expression.

**Figure 8:** Effect of iron/ascorbate and/or BHT treatment on 8-oxoG-DNA Glycosylase levels in Caco-2/15 cells. Caco-2/15 cells were incubated with (0.2 mM/2 mM) FE/ASC and/or (50 µM) BHT for 6 h at 37°C to determine the effects of oxidative stress on 8-oxoG-DNA glycosylase (OGG1) gene expression (A) and protein mass (B). Values are expressed as means ± SEM for three independent experiments carried out in triplicate. ^*^P<0.001.

### Mitochondrial Transcription Factors

Human mitochondrial transcription requires bacteriophage-related RNA polymerase, POLRMT, mtDNA-binding protein, h-mtTFA/TFAM, and two transcription factors/rRNA methyltransferases, h-mtTFB1 and h-mtTFB2. These crucial proteins define mitochondrial biogenesis and gene expression that together likely fine-tune mitochondrial functions. Given the deleterious effects of FE/ASC, it was mandatory to explore how oxidative stress modulates the core protein components required for mitochondrial transcription. PCR and Western Blot analyses showed a significant (P<0.01) increase in mtTFA, mtTFB1 and mtTFB2 gene expression (Figure 9A) and protein mass (Figure 9B) without any changes in POLRMT in Caco-2/15 cells treated with FE/ASC compared with controls. Pre-incubation with BHT attenuated the modifications of those transcription factors.

**Figure 9:** Effect of iron/ascorbate and/or BHT treatment on gene and protein expression of mitochondrial transcription factors in Caco-2/15 cells. Effects of (0.2 mM/2 mM) FE/ASC, (50 µM) BHT or both for 6 h at 37°C on gene expression (**A**) and protein mass (**B**) of mtTFA, mtTB1, mtTB2, POLRMT. A GAPDH cDNA probe was used as a control for RNA loading; β-actin was used as loading control protein. Data originated from three independent experiments. Values are expressed as means ± SEM.^ *^P<0.01.

## Discussion

The Caco-2/15 cell line has been used to examine a variety of intestinal functions. This intestinal model exhibits many of the features of small intestinal epithelial cells. We employed the FE/ASC oxygen radical-generating system to determine how oxidative stress modulates mitochondrial DNA integrity and function in Caco-2/15 cells [20]. Our results show for the first time that FE/ASC can induce lipid peroxidation accompanied by ATP depletion, mitochondrial transport chain complex inhibition, mitochondrial Ca^2+^ overload, cell apoptosis, mitochondrial DNA lesions and mitochondrial transcription factors alterations.

Iron is the most abundant transition metal in mammalian cells and is essential for the physiological function of multiple proteins [42]. However, excess or non-protein-bound (labile) iron can be detrimental because it can initiate oxygen radical formation and promote ROS [43]. Therefore, iron may cause oxidative damage to biological macromolecules and alter the intracellular redox environment, thereby affecting redox-sensitive cell signaling pathways and transcription factors [44], [45]. Although the mechanisms underlying the cytotoxicity of iron in different organs are not fully delineated, many reports have pointed to the participation of iron-mediated peroxidation in numerous pathological states, including atherosclerosis [46], [47], cancer [48], [49], ischemia-reperfusion injury [50], IBD [51], and conditions of iron overload [52]. Several laboratories [19]–[21], [23]–[26], [52]–[54] have shown the ability of iron to initiate strong lipid peroxidation, whereas ascorbic acid can amplify the oxidative potential of iron by promoting metal ion-induced lipid peroxidation. The data presented here clearly indicate that the FE/ASC system functioned as a producer of lipid peroxidation and, at the same time, altered the DNA integrity and the function of mitochondria. It is noteworthy that the iron dose used in the current study is comparable with normal iron concentration in the gut [11]. The deteriorations resulting from the exposure of Caco-2/15 cells to FE/ASC are probably attributable to oxidative stress, because the addition of the BHT antioxidant simultaneously prevented the occurrence of lipid peroxidation and improved the cellular processes of mitochondrial integrity and functions. BHT was selected as an antioxidant because it represents a powerful agent inhibiting iron-mediated oxidative stress and does not have any toxic effects on Caco-2/15 cell culture [21].

Previous reports observed that an accumulation of peroxidation products in mitochondria leads to a decrease in ATP production and compromises the maintenance of cellular homeostasis [55]. In this study, incubation of Caco-2/15 cells with FE/ASC induced a marked decrease in ATP levels. Our data are consistent with previous investigations showing that ATP decreased in the HT-29 intestinal cell-line after oxidative injury by hydrogen peroxide [56]. The fall in ATP synthesis is probably related to the low mitochondrial metabolic activity resulting from the FE/ASC-mediated lipid peroxidation. In fact, electron movement through complexes I, II, III, and IV enables movement of hydrogen ions across the inner membrane into the inter-membrane space creating an electrochemical gradient, which is harnessed into ATP production by ATP synthase in complex V. We reasonably propose that mitochondrial damage from ROS may lead to a degradation in the efficiency of the mitochondrial respiratory chain enzymes and hence a decline in ATP production. The impairment of mitochondrial complex I, II, III and IV activity noted in our experiments may be attributable to ROS-induced cardiolipin damage that has recently been reported in ischemia/reperfusion rat heart, which ultimately led to a decrease in oxidative phosphorylation [57], [58]. The phospholipid cardiolipin is found almost exclusively in the inner mitochondrial membrane where it promotes the optimal function of numerous enzymes involved in mitochondrial energy metabolism. Finally, inactivation of mitochondrial electron transport chain enzymes and/or ATP-synthase may account for the ATP depletion triggered by the administration of FE/ASC to Caco-2/15 cells.

On top of its ATP generation ability, mitochondria also play a part in modulating the amplitude and spatiotemporal organization of Ca^2+^ signals through rapidly accumulating and releasing Ca^2+^ [59], [60]. Indeed, intracellular Ca^2+^ plays a key role in cellular metabolism. However, excessive mitochondrial Ca^2+^ overload can trigger ROS overproduction, mitochondrial membrane depolarization and ATP production inhibition, all hallmark events of mitochondrial dysfunction clearly observed in the present work. Additionally, these defective processes may eventually lead to apoptosis [59], [60], which was also documented in our studies. In particular, mitochondrial Ca^2+^ overload can favor cardiolipin peroxidation, thereby affecting mitochondrial permeability transition, inducing AIF and cytochrome C release, and culminating in mitochondrial dysfunction and apoptosis [61], [62]. Therefore, tools capable of minimizing mitochondrial Ca^2+^ overload would decrease mitochondrial ROS accumulation and improve mitochondrial energy production, which may impact on mitochondrial-oxidative mediated diseases.

The core human mitochondrial transcription machinery comprises a single subunit bacteriophage-related RNA polymerase (POLRMT), mtTFA, and two transcriptional co-activator proteins, h-mtTFB1 and h-mtTFB2. Both factors seem to interact directly with POLRMT forming a heterodimer that, in addition to mtTFA, is required for the accurate initiation on both H_1_ and L promoters [63]. The main function of mtTFA is the maintenance of mtDNA replication and transcription during mitochondria biogenesis [64]. In our study, we observed that mtTFA, mtTFB1, mtTFB2 transcriptional level and protein mass were augmented in the presence of Fe/ASC with no marked difference for POLRMT. Currently, we do not know whether the upregulation of mtTFA, mtTFB1, and mtTFB2 in our experiments represent a compensatory mechanism in response to oxidative stress-related reduction in energy metabolism such as defective electron transport chain, incomplete mitochondrion biogenesis or accelerated apoptosis. Accordingly, mtTFA was found upregulated in response to lipopolysaccharide-induced oxidative damage to mitochondria, presumably to enhance mtDNA levels and OXPHOS activity [65]. Furthermore, over-expression of human TFB2M in HeLa cells induced an increase in TFB1M mRNA levels and protein expression [66], suggesting the existence of a retrograde signaling pathway from mitochondria to the nucleus, which precisely regulates the expression of these related factors. Further investigation is needed to examine these important aspects.

In the present study, FE/ASC raised 8-OHdG that represents one of the most frequently generated oxidative base lesions within DNA, owing to guanine, the lowest redox potential among the nucleic acid bases formed in pathological conditions [67]. Similarly, the double immunofluorescence technique revealed that oxidative DNA damage is induced in colon epithelial cells of the IBD mouse model [68]. Furthermore, nuclei were not affected by FE/ASC-mediated oxidative stress, which confirms that mtDNA is more vulnerable than nuclear DNA to oxidative damage given that it is situated much closer to the site of ROS generation and that mitochondria lack protective histones and far fewer mechanisms that prevent reduced base excision repair activity than DNA from nuclei [69]. Our findings confirm that oxidative DNA damage is one of the most common threats to mitochondrial genome stability.

OGG1 is the DNA repair enzyme that recognizes and excises 8-oxodG [70]. The present study shows that incubation of Caco-2/15 with FE/ASC resulted in a marked decrease in OGG1 transcript level and protein mass. Deficiency in DNA repair enzyme OGG1 has likely important functional consequences, compromising the ability of cells to repair DNA. Therefore, intestinal epithelial cells are as sensitive to lipid peroxidation as other cell types, including kidney cortex cells that accumulate 8-OHdG mainly in the mtDNA and to a lesser extent in nuclear DNA under diabetic conditions [71]. We believe that mtDNA damage is linked to the numerous abnormal processes noted in our study, including ATP generation, Ca^2+^ homeostasis and release of signals for cell death.

In summary, the FE/ASC system in Caco-2/15 appeared to be very effective in promoting lipid peroxidation and, at the same time, altering the mitochondrial function. This mitochondrial dysfunction is probably related to oxidative stress, because the addition of antioxidants prevented the occurrence of lipid peroxidation and improved the mitochondrial function in terms of ATP production, Ca^2+^ homeostasis and apoptotic protein expression. The pattern of our results using the Caco-2/15 cell line may prove useful in elucidating the molecular mechanisms implicated in IBD. Overall, our data suggest that oxidative-mitochondrial dysfunction is not mediated by a single mechanism, but that it may instead be a consequence of multiple vicious circles organized within a complex functional network.
